# Study on the Predictive Value of Thromboelastography in Early Neurological Deterioration in Patients with Primary Acute Cerebral Infarction

**DOI:** 10.1155/2022/4521003

**Published:** 2022-09-25

**Authors:** Xuena Zhang, Xiaohui Jia, Ling Chen, Wenhu Zheng, Jing Zhu, Aiying Ma

**Affiliations:** Department of Internal Medicine, Shanghai Yongci Rehabilitation Hospital, Shanghai 201107, China

## Abstract

**Objective:**

To investigate the predictive value of thromboelastography for the occurrence of early neurological deterioration (END) in patients with primary acute cerebral infarction (ACI).

**Methods:**

150 patients who were hospitalized in the department of neurology of our hospital from September 2020 to September 2021 and were clearly diagnosed with primary ACI by head CT and head magnetic resonance imaging (MRI) were selected and divided into END and non-END groups according to the change in National Institute of Health Stroke Scale (NIHSS) score within 72 h of admission. The general baseline data and laboratory indexes of the first examination at admission were compared between the two groups, and the factors that may affect the occurrence of END were determined by univariate analysis and multivariate logistic regression analysis, and the predictive value of thromboelastography on the occurrence of END after ACI was analyzed by applying the receiver operating characteristic (ROC) curve.

**Results:**

Time to onset, baseline NIHSS score, percentage of diabetes, white blood cell (WBC) levels, C-reactive protein (CRP), and apolipoprotein B (Apo B) levels were higher in the END group than in the non-END group (*P* < 0.05); coagulation reaction time (RT) (3.97 ± 1.16 vs. 5.49 ± 1.03) and kinetic time (KT) (1.32 ± 0.67 vs. 1.82 ± 0.58) were lower in the END group than in the non-END group (*P* < 0.05). Inthe END group (*P* < 0.05) diabetes, baseline NHISS score, CRP level, Apo B level, and RT were independent risk factors for the development of END in patients with ACI (*P* < 0.05). The AUC of RT to predict the occurrence of END in patients with ACI was 0.855 (95% CI: 0784 to 0925, *P* = 0.001), with a sensitivity of 81.70% and specificity of 78.00% when the optimal cut-off value was 0.597.

**Conclusion:**

NIHSS score at admission, CRP, apolipoprotein B, RT shortening, and diabetes mellitus were independent risk factors for the development of END in ACI patients; RT shortening in TEG was predictive of END in ACI patients.

## 1. Preface

Acute cerebral infarct (ACI) is a series of syndromes caused by insufficient blood oxygen supply due to thrombosis, atherosclerosis, and embolism dislodgement in cerebral vessels, which is a common and frequent disease in neurology, with a high incidence, high disability, and a high recurrence rate, and the incidence is getting younger and younger [1, 2]. Early neurological deterioration (END) occurs in 19% to 24% of patients within 72 h after the onset of cerebral infarction and is characterized by progressive worsening of neurological deficits [3, 4]. The occurrence of END often leads to increased length of stay, in-hospital mortality, disability, and a further decline in quality of life, which seriously affects the prognosis of patients [5]. Therefore, early determination of the risk of END occurrence and prediction of its development in ACI patients is beneficial for the identification of high-risk groups and the development of individualized treatment plans such as thrombolysis/anticoagulation to prevent a recurrence, reduce the incidence of END, and promote later recovery.

The pathogenesis of END, which is recognized by most scholars, is mainly divided into two aspects: one is abnormal hemodynamics and the other is abnormal biometabolism [6–8]. Numerous studies [9, 10] have found that END after ACI may be closely related to many clinical and biochemical features such as atrial fibrillation, coronary artery disease, hypertensive cerebral infarction site, low-density lipoprotein cholesterol (LDL-C) concentration, prothrombin time (PT), and D-dimer (D-D). However, there is still a lack of specific marker features that effectively predict the occurrence of early neurological deterioration in patients with acute cerebral infarction, whether considered in terms of clinical manifestations, imaging data, or biochemical index changes. As a thrombotic disease, the coagulation function of patients with ACI has been a research hotspot for neurology/emergency scholars, and a comprehensive and systematic reflection of the coagulation function and fibrinolytic function of the body after acute cerebral infarction is important for predicting the occurrence of END, precise clinical medication guidance, improving the clinical treatment effect, and improving the long-term prognosis of ACI patients [11, 12]. Thromboelastography (TEG) monitors the coagulation process from the whole dynamic process of platelet aggregation, coagulation, and fibrinolysis, which can dynamically reflect coagulation factors, fibrinogen, platelet function, and fibrinolysis, and is a sensitive test for overall evaluation of coagulation, which can provide strong evidence for the existence of the hypercoagulable state in thrombotic diseases [13, 14]. The literature [15] reported that changes in TEG were sensitive predictors of the risk of progression to cerebral infarction in patients with cerebral ischemia and that several of its indicators were positively correlated with the occurrence of cerebral infarction. Based on the above research theories, it is hypothesized that thromboelastography can assess the risk of END by rapidly and comprehensively detecting the coagulation status of patients with ACI. The study intends to analyze the ability of each test index of TEG and traditional coagulation test index to predict the risk of END from the perspective of the development of END in patients with ACI, in order to provide a certain basis for predicting the risk of END after ACI and early intervention treatment.

## 2. Data and Methods

### 2.1. Study Subjects

#### 2.1.1. Source of Subjects

150 patients who were hospitalized in the department of neurology of our hospital from September 2020 to September 2021 and were clearly identified as having primary ACI by head CT and head MRI were consecutively collected. The National Institutes of Health Stroke Scale score (NIHSS) [16] was used to assess the clinical neurological functional status of the patients in this study. In this study, END was defined as an increase in NIHSS score of 2 or more points within 72 h of admission or the development of new neurological deficits, and patients were divided into the END and non-END groups according to the change in NIHSS score. The END group: Patients with ACI had an increase in NIHSS score > or = 2 points within 72 hours of onset. The non-END group: ACI patients with disease severity peaking within 6 hours of onset, no further progression, or stable or gradually improving neurological function after onset.

#### 2.1.2. Inclusion Criteria

(1) All included patients met the diagnostic criteria of ACI [17]; (2) the interval between onset and admission was <24 hours; (3) age >18 years; (4) the admission NIHSS score was less than 16; (5) the diagnosis of ACI was confirmed by head CT + MRI within 24 hours after admission; and (6) the patient or the patient's family agreed to participate in the clinical study and received approval from the hospital medical ethics committee to participate in the trial.

#### 2.1.3. Exclusion Criteria

(1) Transient ischemic attack; (2) cerebral hemorrhage; (3) previous history of cerebral infarction; (4) acute cardiovascular events; (5) patients who were eligible for thrombolysis for intravenous thrombolysis or interventional thrombus retrieval; and (6) patients with lack of clinical data and death during hospitalization.

#### 2.1.4. Data Collection

Clinical data were collected at the time of admission, including gender, age, previous medical history (hypertension, coronary artery disease, diabetes mellitus, and hyperlipidemia), history of smoking and drinking, blood pressure at admission, immediate NIHSS score at admission, first venous blood routine, blood biochemistry, C-reactive protein (CRP), fasting blood glucose (FBG), apolipoprotein A and apolipoprotein B after admission, and head CT + MRI findings within 24 hours of admission. Smokingand alcohol consumption are risk factors according to the relevant WHO definitions and recommendations, a history of smoking: more than 1 cigarette per day for 6 months continuously or cumulatively; a history of alcohol consumption: more than 2 times per week for at least 1 year.

#### 2.1.5. TEG Test

All ACI patients had 5 ml of venous blood drawn from sodium citrate anticoagulation tubes within 24 h of admission for TEG testing (at least 15 min at room temperature before testing), and the equipment used for the test was a YZ5000 thromboelastography, a kit (stored at 2°C to 10°C), and sample cups and lids provided by Shaanxi Yuzeyi Medical Technology Co. The whole procedure of the experiment was carried out in strict accordance with the standard operating procedures of the instrument, and all specimens were tested for TEG within 2 h after collection. The assays include clotting reaction time (RT), maximum amplitude (MA), kinetic time (KT), alpha (*α*) angle, percent lysis at 30 min (LY30), and coagulation index (CI).

### 2.2. Statistical Methods

All experimental data were analyzed and processed using the SPSS 20.0 statistical software. The measurement data were expressed as the mean ± standard deviation (Mean ± SD) if they obeyed normal distribution, and the *t*-test for independent samples was used for comparison between two groups; if the measurement data did not obey normal distribution, they were expressed as median *M* (P25–P75), and the Mann–Whitney U rank sum test was used for comparison between two groups. A logistic regression model was established, with END as the dependent variable, and the relevant univariate variables were included in the multivariate regression analysis. The dominance ratio (OR) and 95% confidence interval (CI) were calculated to analyze the risk factors affecting the development of END in ACI patients with acute cerebral infarction. The difference was statistically significant when *P* < 0.05.

## 3. Results

### 3.1. Comparison of Baseline Data at Admission between the END and Non-END Groups

The analysis of baseline data between the two groups showed that the time of disease onset, baseline NIHSS score, percentage of diabetes mellitus, WBC level, CRP, and apolipoprotein B level was higher in the END group than in the non-END group, with statistically significant differences (*P* < 0.05). There were no statistically significant differences in age, previous hypertension, coronary heart disease, hyperlipidemia, smoking history, alcohol history, baseline diastolic blood pressure (DBP), systolic blood pressure (SBP), white blood cell count (WBC), platelet count (PLT), TC, TG, HDL, LDL, and apolipoprotein A levels between the two groups (*P* > 0.05), and the results are detailed in Table 1.

### 3.2. Comparison of Infarct Sites between the END and Non-END Groups

The site of cerebral infarction was determined based on the report of CT + MRI examination results and imaging images of the patients' heads, and the comparative analysis of different infarct sites (basal ganglia, lobes, brainstem, cerebellum, and corona radiata) between the two groups showed that the differences were not statistically significant (*P* > 0.05).  Table 2.

### 3.3. Comparison of TEG Parameters between the END and Non-END Groups

The analysis of TEG parameters between the two groups showed that the coagulation reaction time RT (3.97 ± 1.16 vs. 5.49 ± 1.03) and kinetic time KT (1.32 ± 0.67 vs. 1.82 ± 0.58) were lower in the END group than in the non-END group, and the differences were statistically significant (*P* < 0.05). The differences were not statistically significant (*P* > 0.05) when comparing the MA, *α*-angle, LY30, and CI between the two groups.  Figure 1.

### 3.4. Logistic Regression Analysis of Risk Factors for the Development of END in ACI Patients

Logistic univariate analysis showed that time to onset, diabetes mellitus, baseline NHISS score, WBC level, CRP level, apolipoprotein B level, RT, and KT were associated with the development of END in ACI patients (*P* < 0.05). Further multiple regression analysis was performed on the indicators that differed in the univariate analysis, and the results showed that diabetes mellitus, baseline NHISS score, CRP level, apolipoprotein B level, and RT were independent risk factors for the development of END in patients with ACI (*P* < 0.05).  Table 3.

### 3.5. Predictive Value of RT for the Occurrence of END in ACI Patients

The ROC curve is shown in Figure 2, and the AUC of RT for predicting the occurrence of END in ACI patients was 0.855 (95% CI: 0784 to 0925, *P*=0.001), indicating that RT has a high degree of predictive value for the occurrence of END, with a sensitivity of 81.70% and a specificity of 78.00% when the optimal cut-off value is 0.597.

## 4. Discussion

Patients with ACI often show clinical manifestations of worsening neurological function in the early stages of the disease, and even through clinical treatment with active thrombolysis, anticoagulation, and symptomatic support, there is still a high lethality and disability rate, and the prognosis of patients is extremely poor [18, 19]. Although there are many studies on the risk factors and mechanisms of ACI-END, there is still a lack of early and effective identification methods, which makes its treatment more difficult, so there is a need to find effective indicators to predict END. There are many studies on ACI and the independent risk factors affecting the development of END after ACI, but the factors that are truly predictive of END after ACI are not well defined, probably due to an incomplete understanding of the underlying pathophysiological mechanisms. The aim of this study is to provide a reference for early targeted control of risk factors and to reduce the incidence of END in ACI patients.

TEG is a coagulation-fibrinolytic system function test that has matured in recent years and is more accurate and comprehensive than conventional laboratory coagulation tests [20, 21]. Recently, some studies have explored the prospect of its application in the diagnosis and treatment of cerebrovascular diseases, such as Elliott et al. [22], who applied TEG to analyze coagulation function in patients with acute cerebral infarction and found that TEG hypercoagulability was prevalent in patients with acute cerebral infarction before thrombolysis compared with normal controls, including shortened RT, increased angle, and shortened KT. In this study, we studied patients with mild to moderate cerebral infarction without intravenous thrombolytic therapy, and the results showed that RT was significantly shorter in TEG in the END group compared to KT in the non-END group (*P* < 0.05), and the findings were consistent with this. In addition, the risk factor logistic regression analysis confirmed that RT shortening was an independent risk factor for the development of END in ACI patients (OR: 1.865, 95% CI: 1.188∼2.906, *P*=0.012), and the ROC curve suggested that the AUC of RT to predict the development of END in ACI patients was 0.855 (95% CI: 0784∼0925, *P*=0.001), with an optimal stage value of 0.597, sensitivity of 81.70% and specificity of 78.00%. RT is the latency period between the placement of the blood sample into the TEG assay and the formation of the first fibrin clot, which represents the combined action of coagulation factors participating in the coagulation initiation process, including endogenous pathways, exogenous pathways, and common pathways, until the fibrin clot begins to form; therefore, RT shortening indicates that the blood is in a hypercoagulable state [23, 24]. The above results suggest that RT may be a better predictor of END in ACI patients, which can be paid attention to during clinical diagnosis or testing to reduce the incidence of END, thus helping patients to restore blood flow early and reducing the probability of adverse prognosis.

In this study, we found that TEG testing was performed in 150 ACI patients centrally, and after correcting for some confounding factors, RT shortening was found to be an independent correlate of whether END occurred, which is useful for predicting END in the clinic. In addition, risk factors such as smoking, diabetes, baseline NHISS, CRP levels, and Apo B should be noted. This study has the following shortcomings: First, the number of patients selected was limited; second, the patient selection excluded patients with moderate to high cerebral infarction, and if more rigorous experimental results are obtained, the scope needs to be expanded for the next study; third, there was no further degree division for the degree of diabetic patients, and the conclusions drawn were not precise enough.

In summary, there are many factors affecting END in patients with acute cerebral infarction, and multifactor logistic regression analysis revealed that NIHSS score at admission, CRP, apolipoprotein B, RT shortening, and diabetes mellitus were independent risk factors for the development of END in patients with ACI. The results of this study suggest that RT shortening of TEG has a certain predictive significance for the development of END in ACI patients, which is of some significance for clinicians to assess the course of cerebral infarction patients at an early stage and take appropriate measures to improve the prognosis of cerebral infarction patients.

## Figures and Tables

**Figure 1:** Comparison of TEG parameters between the END and non-END groups. Note: the comparison of coagulation RT, KT, *α*-angle, coagulation coefficient (CI), maximum clot strength (MA), and percent lysis at 30 min (LY30) between the two groups is shown in the above graphs from (a∼f), respectively. ^*∗*^ indicates *P* < 0.05 compared with the non-END group.

**Figure 2:** ROC plot of the predictive value of RT for the occurrence of END in patients with ACI.

**Table 1:** Comparison of baseline data at admission between the END and non-END groups (*n*, Mean ± SD).

Information		Non-END group (*n* = 109)	END group (*n* = 41)	*t/χ * ^2^	*P*
Gender (*n*, %)	Male	61 (55.96)	26 (63.41)	0.679	0.410
	Female	48 (44.04)	15 (36.59)		

Age (years, Mean ± SD)		62.83 ± 7.67	64.95 ± 7.26	1.530	0.128
Onset of disease (*h*, Mean ± SD)		10.30 ± 2.18	11.17 ± 2.05	2.213	0.028

Hypertension (*n*, %)	Yes	42 (38.53)	19 (46.34)	2.569	0.109
	No	87 (79.82)	22(53.66)		

CHD (*n*, %)	Yes	34 (31.19)	18 (43.90)	2.125	0.145
	No	75 (68.81)	23 (56.10)		

DM (*n*, %)	Yes	23 (21.10)	17 (41.46)	6.317	0.012
	No	86 (78.90)	24 (58.54)		

Hyperlipidemia (*n*, %)	Yes	26 (23.85)	6 (14.63)	1.509	0.219
	No	83 (76.15)	35 (85.37)		

Smoking (*n*, %)	Yes	50 (45.87)	20 (48.78)	0.101	0.750
	No	59 (51.13)	21 (51.22)		

Alcohol consumption (*n*, %)	Yes	33 (30.28)	8 (19.51)	1.738	0.187
	No	76 (69.72)	33 (80.49)		

Baseline SBP (mmHg, Mean ± SD)		151.16 ± 23.38	153.27 ± 24.75	0.485	0.629

Baseline DBP (mmHg, Mean ± SD)		84.81 ± 12.15	85.46 ± 11.80	0.294	0.769

Baseline NHISS score (points, Mean ± SD)		6.53 ± 1.34	9.54 ± 1.87	10.940	0.001

PLT (×10^9^/L, Mean ± SD)		229.75 ± 21.30	230.27 ± 25.44	0.126	0.900

WBC (×10^9^/L, Mean ± SD)		7.19 ± 0.99	8.49 ± 1.23	6.693	0.001

TC (mmol/L, Mean ± SD)		4.43 ± 1.20	4.59 ± 1.21	0.726	0.469

TG (mmol/L, Mean ± SD)		1.80 ± 1.22	1.50 ± 0.79	1.462	0.146

HDL (mmol/L, Mean ± SD)		1.02 ± 0.30	1.08 ± 0.41	0.983	0.328

LDL (mmol/L, Mean ± SD)		2.81 ± 1.10	2.85 ± 1.13	0.197	0.844

CRP (mmol/L, Mean ± SD)		4.78 ± 1.12	6.52 ± 0.76	9.175	0.001

FBG (mmol/L, Mean ± SD)		7.22 ± 0.39	7.26 ± 0.81	0.407	0.685

Apolipoprotein A (g/L, Mean ± SD)		1.21 ± 0.23	1.22 ± 0.21	0.243	0.809

Apolipoprotein B (g/L, Mean ± SD)		0.81 ± 0.14	1.16 ± 0.40	7.963	0.001

**Table 2:** Comparison of infarct sites between the END and non-END groups (*n*, %).

Group/infarct site	Basal ganglia of the thalamus	Lobe of brain	Brainstem	Cerebellum	Corona radiata
Non-END group (*n* = 109)	40 (36.70)	31 (28.44)	26 (23.86)	7 (6.42)	5 (4.59)
END group (*n* = 41)	11 (26.83)	15 (36.59)	8 (19.51)	5 (12.20)	2 (4.88)
*t/χ * ^2^	1.293	0.930	0.320	1.349	0.006
*P*	0.256	0.335	0.571	0.245	0.940

**Table 3:** Logistic regression analysis of risk factors for the occurrence of END in patients with ACI.

Indicators	Single-factor			Multi-factor		
	OR	95% CI	*P*	OR	95% CI	*P*
Onset of disease	1.372	0.749∼2.513	0.230	—	—	—
DM	1.578	1.045∼2.381	0.014	3.435	1.208∼9.764	0.023
Baseline NHISS score	1.669	1.657∼2.389	0.008	2.309	1.457∼3.661	0.010
WBC	1.223	0.854∼1.750	0.350	—	—	—
CRP	3.438	1.407∼8.404	0.001	2.340	1.757∼3.115	0.002
Apolipoprotein B	1.131	1.090∼1.174	0.036	2.040	1.178∼3.532	0.006
RT	1.266	1.082∼1.481	0.003	1.865	1.188∼2.906	0.012
KT	1.670	1.312∼2.126	0.018	1.675	0.626∼4.490	0.523

## Data Availability

The data used to support the findings of the study are available to the corresponding authors upon reasonable request.
